# The role of clustering algorithm-based big data processing in information economy development

**DOI:** 10.1371/journal.pone.0246718

**Published:** 2021-03-11

**Authors:** Hongyan Ma

**Affiliations:** 1 School of Humanities and Social Sciences, Xi’an Jiaotong University, Xi’an, Shaanxi Province, 710049, China; 2 School of Business, Xi’an Fanyi University, Xi’an, Shaanxi Province, 710105, China; Ministry of Natural Resources North Sea Bureau, CHINA

## Abstract

The purposes are to evaluate the Distributed Clustering Algorithm (DCA) applicability in the power system’s big data processing and find the information economic dispatch strategy suitable for new energy consumption in power systems. A two-layer DCA algorithm is proposed based on K-Means Clustering (KMC) and Affinity Propagation (AP) clustering algorithms. Then the incentive Demand Response (DR) is introduced, and the DR flexibility of the user side is analyzed. Finally, the day-ahead dispatch and real-time dispatch schemes are combined, and a multi-period information economic dispatch model is constructed. The algorithm performance is analyzed according to case analyses of new energy consumption. Results demonstrate that the two-layer DCA’s calculation time is 5.23s only, the number of iterations is small, and the classification accuracy rate reaches 0.991. Case 2 corresponding to the proposed model can consume the new energy, and the income of the aggregator can be maximized. In short, the multi-period information economic dispatch model can consume the new energy and meet the DR of the user side.

## Introduction

Big data technology has continued to advance in the late years. As the public gets aware of big data development, big data technology’s development and accumulation are closely connected to people’s daily lives. While improving living standards and quality, big data technology’s development is also accompanied by some problems and challenges [1]. Big data’s rapid development has given birth to a series of new products and new things; simultaneously, it has continuously promoted information economy development. A smart grid, a link in information transmission and information network, is undoubtedly one of the essential information economies’ components. Besides, Demand Side Management (DSM) is a key in developing power information systems [2,3]. However, some traditional data analysis methods become inapplicable given the massive amount of data information in the power information system, requiring searching for new data analysis techniques and methods. The continuous increases in data amount and computational complexity will prolong the calculation time ceaselessly in the power information systems. Therefore, finding a computationally-efficient algorithm tool is imperative. As the information economy develops, researchers have investigated DSM in the power information systems. Bazydlo and Wermiriski (2018) addressed the increasing power demand problems in power information systems and proposed a method to reduce the peak load using the home Local Area Network (LAN) system [4]. Yang and Xia (2017) proposed a power system for the DSM of household Photovoltaic (PV) hybrid power systems under Time-Of-Use (TOU) electricity prices. This system combined the power dispatch layer and the home appliance dispatch layer, showing significant advantages in reducing grid energy consumption [5]. Hamidpour et al. (2019) proposed a resource planning method for power systems to coordinate the expansion planning of power generation and transmission under Demand Response (DR) [6]. Apparently, investigations on DSM in power systems are various.

Given rapid data growth and development, correctly classifying different data types is necessary. While classifying and arranging data, clustering is a useful data analysis technique, which belongs to the category of unsupervised learning [7,8]. Unsupervised learning refers to extracting regular attributes from the initial data that have never been labeled. The cluster analysis method classifies data via the correspondence between data; the greater the similarity between the data, the better the corresponding cluster analysis effect [9,10]. Applying cluster analysis methods to process and classify big data may be a feasible method for power information systems with massive amounts of data. Hence, cluster analysis methods have been applied to power systems. Ma et al. (2019) studied the multi-level railway power conditioner based on power quality management of high-speed traction systems; the system’s dynamic performance was improved based on equivalent analysis of equivalent mathematical models [11]. Regarding the power system’s inertial frequency response, Lara-Jimenez et al. (2017) proposed a method to identify generator groups that formed inertial response clusters and proved its effectiveness given network topology changes and interference [12]. In summary, many fruitful results in applying cluster analysis methods to power systems are achieved. Nevertheless, research on applying this data method to analyze user-side DR is rarely reported.

In this regard, the clustering analysis is combined with user-side DR creatively to explore the effectiveness of clustering analysis in power network system users and analyze the information economic dispatch method applicable in DR. Furthermore, the Distributed Clustering Analysis (DCA) method and multi-period information economic dispatch model are introduced, in an effort to provide a reference for big data processing in power information systems.

## Methods

### Two-layer DCA

The rapid development of computer information technology and its big data technology has provided adequate support and prerequisites for improving the informationization level of smart grids. While smart grids are developing, the user side accumulates many electricity consumption data and information. Hence, mining the hidden information from these data is of great significance for improving the quality of service and promoting the utilization of energy under information economy development [13,14]. On this basis, seeking an appropriate data processing method is useful in providing decision-making support for enterprises and processing and solving a series of difficult problems. Here, processing power load data is the premise of the information economy. The global and local data and information transmission are considered to propose a two-layer framework based on DCA. The details are shown in Fig 1 below.

**Fig 1:** Two-layer framework based on DCA.

The DCA-based framework system embodies three calculation levels: decomposition, clustering, and merging. The decomposition calculation primarily decomposes a site into smaller and independent sub-data. The clustering calculation aims to cluster the sub-data obtained by decomposition in a local area so that the secondary clustering can be performed on this basis. The merging calculation applies complicated and stable clustering algorithm tools to achieve secondary clustering of representative data depending on the above clustering results. Overall, the clustering framework is formed by local and global clustering; more straightforward algorithm tools can obtain clustering results for the former. For the latter, complicated and stable algorithm tools are needed to make the final clustering more accurate. Therefore, the local clustering method in the clustering framework is the K-Means Clustering (KMC) algorithm. For the global clustering in the clustering framework, the complicated Affinity Propagation (AP) algorithm is utilized.

#### (1) Optimization of KMC algorithm

KMC is a typical clustering algorithm. This algorithm can process batch data rapidly. However, the traditional KMC algorithm is sensitive to the starting clustering center and requires manual determination in the clustering process, reducing the accuracy of final clustering results [15,16]. According to these problems in the traditional KMC algorithm, the SSE (Sum of Squares due to Error) index [17] is introduced, and the distance is improved. The equation expression corresponding to the adjusted distance *D* is:

$$D={\sum_{i=1}^{n}\left[\lambda_{i}^{\prime }\left(F_{t}-C_{j}\right)\right]}^{2}+\sum_{k=1}^{n}\lambda_{k}{\left(F^{\prime }-C_{j}^{\prime }\right)}^{2}$$ (1)

In (1), *F*_*t*_ represents the time domain’s feature set, *F*’ represents other feature sets, *C*_*j*_ and $C_{j}^{\prime }$ denote the feature sets of the cluster center, $\lambda_{i}^{\prime }$ and *λ*_*k*_ denote the weight, *i* and *k* stand for the data points in the algorithm. *n* refers to the total number of data points. The equation in which the Square Sum of Error (SSE) index is introduced is:

$$SSE={\sum \left(x-C_{j}\right)}^{2}$$ (2)

In (2), *x* represents the independent variable. Conditions of obtaining clusters’ optimal number for local clustering in the framework are:

$$SSE-SSE_{new}<5$$ (3)

#### (2) Optimization of the AP algorithm

Among various clustering algorithms, the AP algorithm’s essence is partition [18]. In this algorithm, the equations for attracting information matrix *R* and attribution information matrix *A* are expressed as:

$$R\left(i,k\right)=s\left(i,k\right)-\underset{k^{\prime }\neq k}{\max}\left\{a_{t}\left(i,k\prime \right)\right\}$$ (4)

$$A_{t+1}\left(i,k\right)=\min\left(0,R_{t}\left(k,k\right)+\sum_{i^{\prime }\notin \left(i,k\right)}\max\left\{0,R_{t}\left(i^{\prime },k\right)\right\}\right),i\neq k$$ (5)

$$A_{t+1}\left(k,k\right)=\sum_{i^{\prime }\neq k}\max\left\{0,R_{t}\left(i^{\prime },k\right)\right\}$$ (6)

In (4), (5), and (6), *i* and *k* represent data points, *s*(*i*,*k*) represents the similarity between *i* and *k*, *R*(*i*,*k*) stands for the attraction information in the information matrix, i.e., the element, *A*(*i*,*k*) stands for the attribution information, and *t* corresponds to the current value. On this basis, the damping coefficient *ϑ* is introduced to update the element values in *R* and *A* to optimize the algorithm’s convergence performance. The corresponding equations are:

$$R_{t+1}^{\prime }\left(i,k\right)=\vartheta \cdot R_{t}\left(i,k\right)+\left(1-\vartheta \right)\cdot R_{t+1}\left(i,k\right)$$ (7)

$$A_{t+1}^{\prime }\left(i,k\right)=\vartheta \cdot A_{t}\left(i,k\right)+\left(1-\vartheta \right)\cdot A_{t+1}\left(i,k\right)$$ (8)

In (7) and (8), $R_{t+1}^{\prime }\left(i,k\right)$ refers to the updated element, and $A_{t+1}^{\prime }\left(i,k\right)$ stands for the updated attribution information.

The weights of time-domain features in the global situation are not updated to distinguish the electrical load conditions under different local sites. Instead, the data features corresponding to the local sites are considered. On this basis, the equation for similarity matrix *s* update processing is expressed as:

$$s\left(i,j\right)=\sum_{i=1}^{n}{\left(d_{i}-d_{j}\right)}^{2},i\neq j$$ (9)

In (9), *d*_*i*_ and *d*_*j*_ represent the preferred feature sets corresponding to the load curves *x*_*i*_ and *x*_*j*_.

### User-based DR flexibility

Under the big data environment, processing the information in the smart grid has changed dramatically. From the users’ perspective, electric energy consumption has changed from the traditional passive acceptance to the current active participation. The DR flexibility analysis on the user side is of great significance based on the new information on energy consumption in the power grid. It can accurately judge the flexibility shown by the user side, thereby improving the information energy consumption, playing a vital role in optimizing and adjusting the entire power information system and the relevant resources and energy in the power system [19,20]. While analyzing the DR flexibility, crucial factors include power consumption level, power consumption stability, power consumption tendency, and load changes. Functionally, some of the above factors can play a positive role in DR, while some cannot. In DCA, cluster centers characterize the stability of electricity load; for this feature, user entropy *E*_*u*_ can be used for analysis, and the corresponding equation expression is:

$$E_{u}=\sum_{i=1}^{w}L_{i}\log_{2}L_{i}$$ (10)

In (10), *L*_*i*_ represents the *i*-th load characteristic, and *L* corresponds to the load. The smaller the *E*_*u*_, the more the information in the entire power system, and the more stable the system state. *w* corresponds to the adjustment coefficient. On this basis, the equation for DR flexibility analysis on the user side is expressed as:

$$DL_{l}=\sum_{i=1}^{n_{f}-1}\tau_{i}F_{i}-\tau_{u}E_{u}$$ (11)

$$DL_{u}=\sum_{i=1}^{n_{f}-1}\tau_{i}F_{i}+\tau_{u}E_{u}$$ (12)

In (11) and (12), *F*_*i*_ represents the *i*-th load characteristic index, *τ*_*i*_ is the corresponding weight, *τ*_*u*_ represents the weight based on *E*_*u*_, and *DL*_*l*_ represents the price-based DR flexibility on the user side, and *DL*_*l*_ is the incentive DR flexibility on the user-side. A more considerable value of DR flexibility shows that this type is more applicable in DR flexibility analysis. Power information systems contain many users based on the aggregator. Hence, analyzing the behavior characteristics of all users is challenging. Here, DCA is applied to classify users, which analyzes the overall behavioral characteristics of all users. Flexibility analysis under the aggregator can be calculated using (13) and (14) combined with the above user-side flexibility analysis calculation.

$$DL_{{}_{la}}=\frac{\sum_{i=1}^{u}n_{ui}DL_{li}}{n_{LA}}$$ (13)

$$DL_{{}_{ua}}=\frac{\sum_{i=1}^{u}n_{ui}DL_{ui}}{n_{LA}}$$ (14)

In (13) and (14), *DL*_*la*_ and *DL*_*ua*_ respectively represent price-based flexibility and incentive-based flexibility under the aggregator, *n*_*ui*_ stands for the number of users under the class *i*, and *n*_*LA*_ represents the total number of users based on the aggregator. Among the two different DR types, i.e., the price type and the incentive type, the latter is more useful in reflecting user wishes. Therefore, the incentive type is chosen for the information dispatch strategy in the following analysis on user-side DR flexibility.

### Construction of multi-period information economic dispatch model

A smart grid, an information system with a massive amount of data, is challenging to dispatch loads directly. Therefore, a grid system that can integrate resource information, a load aggregator that can meet the power demand on the user side, and the primary users of electric power consumption is considered. According to the above analysis on the user-side DR flexibility in the power information system, the load aggregator is chosen as the research subject. The new information energy’s incentive electricity price is applied to construct the smart grid’s information dispatch strategy. In this distributed smart grid information dispatch framework, the fundamental structural layers are smart grid information dispatch, aggregator decision-making, and load response. The primary role of smart grid information dispatch aims to issue information dispatch tasks. In smart grid systems, distributed new energy and interconnected grid transmission are the principal ways to obtain electric power. The aggregator decision-making layer aims at the interaction between the power grid information system and users and dispatches the dispatchable capacity and plan in the information system. The load response layer can receive information dispatch signals, which depend on intelligent information terminals to collect electricity consumption information. Its principal function is to implement dispatch tasks. Information dispatch includes day-ahead dispatch and real-time dispatch. The former is cleared before the day, and the latter is cleared every hour. On this basis, the implementation process of information economic dispatch under this multi-period is shown in Fig 2 below.

**Fig 2:** Implementation process of information economic dispatch in multi-periods.

In this multi-period information economic dispatch framework, users respond to dispatching instructions depending on load regulation. Due to the large differences between residential users, it is only ideal for aggregators to analyze the use of all home appliances. Thus, aggregators must understand the electricity consumption of relevant residents. According to the differences in the use time, the use of electrical appliances can be divided into three load types: uncontrollable, translatable, and interruptible loads. The last load type can achieve load reduction. The dispatch model constraints based on this load can be described as:

$$C_{il\min}*P_{il\_t}\leq C_{il\_t}\leq C_{il\max}*P_{il\_t}$$ (15)

$$P_{il\_t}\in \left\{0,1\right\},\forall t\in T_{il}$$ (16)

$$P_{il\_t}=0,\forall t\notin T_{il}$$ (17)

In (15)–(17), *C*_*il*_*t*_ represents the interruptible load at time *t*, *C*_*il*max_ corresponds to the upper limit, *C*_*il*min_ corresponds to the lower limit, *P*_*il*_*t*_ refers to the number of reductions, and *T*_*il*_ stands for the dispatch contract period. Furthermore, the electricity consumption level of residential users corresponding to aggregator *n* can be expressed as:

$$Q_{i}^{n}=\sum_{t=1}^{T}\left(C_{fix\_t}+C_{ddl\_t}-C_{il\_t}\right)$$ (18)

In (18), $Q_{i}^{n}$ represents the electricity consumption reported by residential users, *C*_*fix*_*t*_ denotes the electricity consumption of uncontrollable loads, *C*_*ddl*_*t*_ refers to the total electricity consumption corresponding to time *t*, and *C*_*il*_*t*_ stands for the interruptible load. Only the revenue corresponding to the aggregator is considered during the dispatching process. In the day-ahead dispatch, the aggregator reports the schedulable capacity based on its flexibility. The load aggregator aims to obtain the maximum profit. The equation for the objective function corresponding to this is expressed as:

$$\max B=\left(1+DC_{ca}^{n}\right)*\sum_{i\in T}C_{i\_incentive}*Q_{i}^{n}-C_{penalty}*\sum_{i\in T-1}Q_{i\_T-1}^{n}$$ (19)

In (19), *C*_*i_incentive*_ refers to the incentive price of new energy corresponding to the dispatch period *T*, *C*_*penalty*_ represents the penalty price, $DC_{ca}^{n}$ denotes the flexibility of the aggregator’s DR, and $Q_{i\_T-1}^{n}$ represents the default electricity. The incentive electricity price is set as:

$$C_{i\_incentive}=-\alpha_{j}\sum_{n=1}^{N}Q_{i}^{n}+\beta$$ (20)

$$\alpha_{j}=\alpha_{j-1}+\frac{\max\left(Q_{i}^{n}-Q_{cv}\right)}{\sum_{t\in T}\left|Q_{i}^{n}-Q_{cv}\right|}$$ (21)

In (20) and (21), *α* represents a correction factor, *β* corresponds to a constant, and *Q*_*cv*_ stands for new energy output. In the real-time dispatching process, the resident users use electricity following the signed contract, and the default electricity *ξ* of the resident users is regarded as subject to a truncated normal distribution. The corresponding probability density function is:

$$f\left(\xi ,\mu_{\xi },\sigma_{\xi },\xi_{1},\xi_{u}\right)=\{\begin{array}{c} \varphi \left(\frac{\xi -\mu_{\xi }}{\sigma_{\xi }}\right)\\ \sigma \left[\Phi \left(\frac{\xi_{u}-\mu_{\xi }}{\sigma_{\xi }}\right)-\Phi \left(\frac{\xi_{1}-\mu_{\xi }}{\sigma_{\xi }}\right)\right]\\ 0 \end{array}$$ (22)

In (22), *φ* denotes the probability density function, Φ signifies the cumulative distribution function; corresponding to the density function, *ξ* refers to the independent variable, *μ*_*ξ*_ stands for the mean, and *σ*_*ξ*_ denotes the standard deviation. Then the default electricity expectations of residents can be obtained:

$$E\left(\xi \right)=\kappa q^{'}\frac{\varphi \left(0\right)-\varphi \left(\frac{1}{\kappa }\right)}{\Phi \left(\frac{1}{\kappa }\right)-\Phi \left(0\right)}$$ (23)

$$\mu_{\xi }=0,\sigma_{\xi }=\kappa q^{'}$$ (24)

In (23) and (24), *q* represents the default electricity of residential users, and *κ* represents a coefficient that can reveal the differences between different residential users. Finally, the equation corresponding to the default rate *W*_*b*_ can be expressed as:

$$W_{b}=\frac{\sum_{i\in N}q_{i}}{Q_{i}^{n}}$$ (25)

The revenue corresponding to the aggregator can be expressed as:

$$\max B=\sum_{t\in T}\left(\sum_{i\in n}Q_{i}^{nr}*C_{r\_t}-\sum_{i\in n}Q_{i}^{C\_t}*C_{C\_t}\right)$$ (26)

In (26), $Q_{i}^{nr}$ represents the decision variable, *C*_*r*_*t*_ denotes the real-time electricity price, $Q_{i}^{C\_t}$ refers to the electricity purchased by the aggregator from the grid, and *C*_C_*t*_ stands for the price of electricity purchased and sold.

### Algorithm performance and case analyses

According to the literature, two local sites are set up to evaluate the proposed two-layer DCA’s performance; each site contains 1000 load curves. For local clustering, time domain and volatility indexes are introduced to reduce data dimensionality. For global clustering, time domain and frequency domain indexes are introduced to reduce data dimensionality. According to indexes such as Davies-Bouldin (DB) index, classification accuracy, iteration times, and calculation time, several classic algorithms are introduced to test the performance of the two-layer DCA proposed above, including the centralized KMC algorithm (K) [21], the centralized AP algorithm (AP) [22], the K-means-AP clustering algorithm based on time-domain features (TK-AP), and the distributed K-means-AP clustering algorithm based on optimum combined features (CK-AP). The proposed algorithm’s effectiveness is tested by comparing various indexes. Also, the clustering results of different algorithms are compared and analyzed to evaluate the algorithms’ performance.

The effectiveness of the multi-period information economic dispatch model constructed above is verified by modifying the IEEE 33 power node system. This case analysis sets four aggregators. The correspondence between jurisdiction nodes and aggregators in the IEEE 33 system is shown in Table 1 below. For real-time dispatch, this case analysis assumes that the default rate of users is 22%. The new information energy consumption corresponding to different aggregators is analyzed according to the above two-layer DCA. Expressly, the two cases are set as follows:

Case 1: The aggregator optimized the day-ahead dispatch scheme, as shown in Eq (19).
Case 2: Aggregators use the proposed multi-period information economic dispatch model based on day-ahead dispatch and real-time dispatch.

**Table 1:** Parameter settings of power information economic dispatch based on aggregator optimization.

Aggregators	A	B	C	D
Flexibility	0.56	0.53	0.42	0.47
Jurisdiction nodes	1–9	10–17	18–26	27–33

## Results and discussion

### DCA’s performance

According to the DB index, the performance comparison results of several algorithms, classification accuracy, iteration times, and calculation time are shown in Fig 3 below.

**Fig 3:** Comparison of several algorithms’ performances.

Compared with the centralized algorithms, distributed clustering algorithms’ calculation time is lessened. For example, the calculation time required by the centralized KMC algorithm and the AP algorithm is 9.23s and 9.51s, respectively. Nevertheless, the calculation time required by several distributed clustering algorithms is lessened significantly. In particular, the calculation time required by the proposed DCA is only 5.23s. Furthermore, the algorithm proposed has the least iteration times and the smallest value of the DB index. Its classification accuracy can reach 0.991. In general, the proposed two-layer DCA has the best performance.

The comparison between the centralized KMC algorithm and the centralized AP algorithm, as well as the clustering results of the algorithm proposed based on user power consumption, is shown in Fig 4 below.

**Fig 4:** Clustering results of centralized clustering algorithms and proposed DCA.

The above analyses demonstrate that the calculation time required by the proposed DCA is short, which is more applicable to process big data. Because the smart grid is an information system with a massive amount of data, applying DCA is obviously advantageous. The above performance comparison of different algorithms suggests that if the amount of data in the information system is the same, for DCA, the AP algorithm has a more prolonged time consumption than the KMC algorithm, which may correlate to the algorithms’ complexity. The applicability shown by DCA is high in the data processing based on the smart grid. The two-layer DCA proposed has the least iteration times. This index also explains the excellent performance of the clustering algorithm in terms of calculation time. It reflects from the side that the DCA proposed can optimize the clustering convergence performance of the simulated data, thereby presenting the best clustering results. Jasinski et al. (2019) adopted cluster analysis to evaluate the distributed power generation and grid consumption [23]. They found that cluster analysis showed good applicability in automatically identifying relevant events in the power system, providing adequate support to the results obtained.

### Case analyses and comparison of information economic dispatch model

Under Case 1 and Case 2, the new energy consumption situation of the power information system corresponding to the four aggregators is shown in Fig 5 below.

**Fig 5:** New energy consumption situation of the power information system based on Case 1 and Case 2.

In case 1, the aggregator adopts an optimized dispatch strategy based on the incentive electricity price, which can process the new energy consumption. In contrast, in Case 2, corresponding to the information economic dispatch model proposed, the electricity consumption generated during the PV output period is higher than the electricity consumption in Case 1, such as the period from 10:00 to 14:00.

The comparison results of incentive electricity prices based on Case 1 and Case 2 are shown in Fig 6 below.

**Fig 6:** Comparison results of incentive electricity prices based on Case 1 and Case 2.

In both Case 1 and Case 2, the corresponding incentive electricity price is consistent with the real-time electricity price during the valid period of PV output. On the contrary, outside this valid period, from 10:00 to 14:00, the incentive electricity price in Case 2 is higher than that in Case 1.

The comparison results corresponding to the four aggregators’ revenue based on Case 1 and Case 2 are shown in Fig 7 below.

**Fig 7:** Comparison of aggregators’ revenue based on Case 1 and Case 2.

Compared with Case 1, the corresponding revenue of the four aggregators in Case 2 has increased significantly. For example, compared with Case 1, the revenue of Aggregator 1 in Case 2 has increased by 139.36%. The revenue of Aggregator 2 in Case 2 has increased by 168.44%. The revenue of Aggregator 3 in Case 2 has increased by 190.31%. The revenue of Aggregator 4 in Case 2 has increased by 228.03%.

The above results demonstrate that the multi-period information economic dispatch model constructed considers the user default and the uncertainty of PV output in new energy consumption, realizing real-time information dispatch. According to the different real-time changes in PV output, applying the proposed multi-period information economic dispatch model to Case 2 can adjust electricity consumption in real-time. For the new energy consumption in the power information system, the aggregator maximizes its revenue as a prerequisite so that the quoted electricity price is increased, increasing the incentive electricity price to some extent. According to the fluctuations in incentive electricity prices corresponding to different aggregators, the electricity consumption behavior of the aggregators in both cases can consume new energy in the power information system, which also shows that the active participation of aggregators in the consumption of new energy has a particular impact on promoting the setting of incentive electricity prices. The aggregators have maximized the revenue goals in Case 2 under the dual effects of day-ahead dispatch and real-time dispatch. In general, the multi-period information economic dispatch strategy based on the two-layer DCA proposed can improve the new energy consumption and positively affects the power dispatch planed by the aggregators based on their actual situations. Le et al. (2020) applied the KMC algorithm to the daily load demand analysis of the power system. They found that this method positively affected cost savings in the power system [24]. KMC algorithm is also employed in the proposed two-layer DCA algorithm, which further confirms the applicability of clustering analysis in power systems.

## Conclusions

The user-side DR flexibility in the smart grid system is analyzed based on the proposed DCA and multi-period information economic dispatch model. Results find that DCA has higher applicability than the centralized clustering algorithms in the cluster analysis of batch big data problem, which also shows a high classification accuracy. The multi-period information economic dispatch model can significantly promote the new energy consumption in the power information system and maximize the revenue goals of the aggregators in real-time dispatch. Case 2 corresponding to the proposed model shows good performance in the consumption of new energy. The aggregator can maximize the revenue target, and the incentive electricity price is higher than that in Case 1. The research results can provide some data support and a reference for the economic operation of the smart grid systems under the background of big data. The cluster analysis method is applied to analyze user-side DR flexibility in the smart grid system creatively, positively affecting the application scope of big data analysis.

As the information economy develops speedily, DR based on the regional energy network covers multiple areas. Although some useful information is obtained, the following problems are found: (1) in the framework of two-layer DCA, local sites are partitioned randomly, and the types of algorithms selected in the performance comparison are limited. The following work will deepen the exploration of combined optimization algorithms to build more efficient algorithm tools in processing batch power data. (2) The multi-period information economic dispatch model is built on DCA. Nevertheless, the model is currently not applicable to large-scale power systems. Therefore, the information economic dispatch model will be further optimized and constructed to build a system applicable in a complicated dispatch environment, which is also a direction for future improvement and efforts.

## Supporting information

S1 Data (XLS)
